The article "A Machine Learning Approach Using XGBoost Predicts Lung Metastasis in Patients with Ovarian Cancer" was published in 2022. Journal: Biomed Res Int.

# A Machine Learning Approach Using XGBoost Predicts Lung Metastasis in Patients with Ovarian Cancer

**DOI:** 10.1155/2022/8501819

**Published:** 2022-10-12

**Authors:** Yufei Yuan, Ruoran Wang, Mingyue Luo, Yidan Zhang, Fanfan Guo, Guiqin Bai, Yang Yang, JingZhao

**Affiliations:** ^1^Xi'an People's Hospital (Xi'an Fourth Hospital), Xi'an, Shaanxi, China; ^2^Department of Neurosurgery, West China Hospital, Sichuan University, Chengdu, Sichuan, China; ^3^Northwest Women and Children's Hospital, Shaanxi, China; ^4^The First Affiliated Hospital of Xi'an Jiaotong University, Shaanxi, China

## Abstract

**Background:**

Liver metastasis (LM) is an independent risk factor that affects the prognosis of patients with ovarian cancer; however, there is still a lack of prediction. This study developed a limit gradient enhancement (XGBoost) to predict the risk of lung metastasis in newly diagnosed patients with ovarian cancer, thereby improving prediction efficiency. *Patients and Methods*. Data of patients diagnosed with ovarian cancer in the Surveillance, Epidemiology, and Final Results (SEER) database from 2010 to 2015 were retrospectively collected. The XGBoost algorithm was used to establish a lung metastasis model for patients with ovarian cancer. The performance of the predictive model was tested by the area under the curve (AUC) of the receiver operating characteristic curve (ROC).

**Results:**

The results of the XGBoost algorithm showed that the top five important factors were age, laterality, histological type, grade, and marital status. XGBoost showed good discriminative ability, with an AUC of 0.843. Accuracy, sensitivity, and specificity were 0.982, 1.000, and 0.686, respectively.

**Conclusion:**

This study is the first to develop a machine-learning-based prediction model for lung metastasis in patients with ovarian cancer. The prediction model based on the XGBoost algorithm has a higher accuracy rate than traditional logistic regression and can be used to predict the risk of lung metastasis in newly diagnosed patients with ovarian cancer.

## 1. Introduction

Ovarian cancer is the fifth leading cause of cancer-related death in women [1]. Most patients are already at an advanced stage since there are no evident symptoms in the early stages, and 70% of patients with advanced cancer already have distant metastases at the time of diagnosis [2]. Ovarian cancer can spread through intraperitoneal, lymphatic, and blood transmission routes [3]. The most common distant metastasis site is the liver, followed by the distant lymph nodes, lungs, bones, and brain. Distant metastasis is associated with poor overall survival. Patients with lung metastases have the worst survival prognosis [4]. Pneumonectomy for specific patients is safe and effective [5]. Therefore, developing predictive models to predict lung metastasis can help guide clinical strategies, which is important for improving the prognosis of patients with ovarian cancer.

At present, there have been several population-based large data studies on ovarian cancer, but most of them focus on the risk factors for ovarian cancer survival and prediction model construction [6–8]. Although studies have performed univariate and multivariate logistic regression analyses to determine the factors related to the development of epithelial and serous ovarian cancer lung metastasis [9, 10] and build models and nomograms to predict the risk of lung metastasis in patients with ovarian cancer [11], the C-index was 0.761 (0.736-0.787), and the accuracy was not high. To a certain extent, these prediction models still have shortcomings, such as insufficient prognostic strength, large fluctuation range, and poor stability. A standardized assessment of the risk of lung metastasis in patients with ovarian cancer is still lacking. Machine learning can transform measurement results into relevant predictive models, especially cancer models, based on the rapid development of large datasets and deep learning [12]. Previous studies have proposed a novel boundary-constrained network (BCNet) for accurate polyp segmentation [13]. However, most models are based on traditional ML algorithms created in the last century, including backpropagation neural networks (BPNN), multilayer perceptrons (MLP), decision trees, support vector machines (SVM), and Bayesian networks [14]. Compared to traditional ML algorithms, the eXtreme Gradient Boosting (XGBoost) algorithm, which was first released in 2016, is more novel and complex. XGBoost is a large-scale machine learning algorithm. This is an improvement over gradient-boosted decision trees (GBDT). A single decision tree is a simple and weak classifier. However, ensemble models of trees, such as random forest [15] and GBDT [16], can be much better. Compared with GBDT, XGBoost uses a technique called “feature subsampling,” which is used in random forests to prevent overfitting. XGBoost is more novel and complex compared to traditional ML algorithms. An important advantage of XGBoost over traditional ML algorithms is that it has random seeds, which can improve the model by repeating operations even if the parameters remain unchanged. It can handle missing data efficiently and flexibly and assemble weak prediction models to build accurate predictions. It has a better performance in terms of the calculation speed [17]. In contrast, SVMs are not good at dealing with problems with a large number of samples and variables, whereas Bayesian networks are easy to train quickly but are not sufficiently complex [14]. Many studies have shown that XGBoost is more suitable for predicting the large data volume of the SEER database than other machine learning methods. XGBoost has the best performance in predicting lymph node metastasis in oral squamous cell carcinoma and prostate cancer and survival in esophageal cancer [18–20].

Our goal was to develop a new decision-support ML model based on big data to predict the risk of lung metastasis in patients with ovarian cancer. This study is the first to develop a machine-learning-based prediction model, XGBoost, for lung metastasis in patients with ovarian cancer. This study is aimed at verifying XGBoost's predictive value for lung metastasis in patients with ovarian cancer and improving the prediction efficiency of lung metastasis in patients with ovarian cancer to better guide clinical strategies.

## 2. Patients and Methods

### 2.1. Study Population

Data were obtained from the Surveillance, Epidemiology, and End Results (SEER) database. The SEER ^∗^Stat 8.3.5 software (https://seer.cancer.gov/data/) was used to access the database. The site code was restricted to the ovary (International Classification of Diseases for Oncology-3/WHO 2008). Since the details of metastases were not recorded before 2010, patients with primary ovarian cancer aged ≥ 18 years at diagnosis and between 2010 and 2015 were analyzed. The exclusion criteria for patient selection were as follows: (1) unknown grade; (2) unknown AJCC T, N stage, and AJCC T0 stage; (3) unknown metastasis information; (4) unknown tumor size; (5) unknown laterality; and (6) unknown therapy information (Figure 1). This study enrolled 16059 patients with ovarian cancer based on the inclusion and exclusion criteria. Data regarding clinical characteristics, including age, race, marital status, insurance status, year of diagnosis, histological type, grade, laterality, clinical AJCC T, N stage, tumor size, metastatic status, and therapy information, were collected from the SEER database. Informed consent was not required to use SEER data since all information has been identified, and no personal identifying information was used in this analysis. This study analyzed 13 clinical and pathological features. Variables that could be used for further analysis included age, race, marital status, insurance status, tumor size, laterality, grade, TNM staging (AJCC 7th edition), tumor metastasis location, and histological classification. In the SEER database, several methods have been introduced to define race. We also redefined race as white, black, and others (American Indian/AK Aborigines and Asian/Pacific Islanders). The grade was defined as undifferentiated, low-, medium-, or well-differentiated. Insurance is defined as insured or uninsured. Marital status was defined as being married, unmarried, or separated. Tumor size was defined as <2 cm, 2-5 cm, and >5 cm. Laterality was defined as left, right, or bilateral. All variables were defined as categorical variables, and the study complied with the 1964 Helsinki Declaration and its later amendments or comparable ethical standards.

### 2.2. Statistical Analysis

The SPSS 21 software was used for statistical analysis. Categorical data are expressed as frequency (%) and were analyzed using the chi-square test. The Kolmogorov-Smirnov test was used to verify the normality of the variables. Normally distributed variables are expressed as mean ± standard deviation, whereas nonnormally distributed variables are expressed as median (interquartile range). Student's *t*-test and Mann–Whitney *U* test were used to compare continuous variables that were normally or nonnormally distributed. The chi-square test or Fisher's exact test was used to compare categorical variables, and our prediction model was based on XGBoost, which is a scalable tree-boosting system. The model used the training set for training and validation set for testing to determine its accuracy. In our prediction model, the number of ensemble decision trees was 60, and the maximum depth of each tree was 15. This was calculated through repeated attempts to obtain the best accuracy and avoid overfitting. We implemented the XGBoost model to analyze each variable's contribution to lung metastasis in ovarian cancer. After identifying the variables through XGBoost, we used them to build the XGBoost algorithm model. The result of XGBoost is a continuous output between 0 and 1, representing the probability of lung metastasis in patients with ovarian cancer. We tested the predictive model's performance using the area under the curve (AUC) of the receiver operating characteristic (ROC) curve.

## 3. Results

### 3.1. Characteristics of the Study Population

According to the inclusion and exclusion criteria, 16,059 of the 35,333 patients with ovarian disease registered between 2010 and 2015 were collected from the SEER database. The basic information of the patients is listed in Table 1. The median age of patients with lung metastasis was higher than those without lung metastasis (62 vs. 59, *P* < 0.01). Compared with patients without lung metastasis, there were no significant differences in race (*P* = 0.192), marital status (*P* = 0.170), insurance status (*P* = 0.932), tumor size (*P* = 0.139), or brain metastasis (*P* = 0.017) in patients with lung metastasis. Significant differences were observed in tumor laterality (*P* < 0.001), tumor grade (*P* < 0.001), AJCC T stage (*P* < 0.001), AJCC N stage (*P* < 0.001), bone metastasis (*P* < 0.001), liver metastasis (*P* < 0.001), and histological type (*P* < 0.001) between the two groups.

### 3.2. Construction and Evaluation of the Prediction Models Based on XGBoost

The gbm (Light Gradient Boosting Machine) algorithm results (Figure 2) showed that the top five important factors were age, laterality, histological type, grade, and marital status. Receiver operating characteristic (ROC) curves were plotted (Figure 3). XGBoost showed good discriminative ability, with an AUC of 0.843. Accuracy, sensitivity, and specificity were 0.982, 1.000, and 0.686, respectively.

## 4. Discussion

The incubation period from the diagnosis of ovarian cancer to the development of lung metastasis can be as long as 108 months [21]. Routine imaging tests such as computed tomography (CT) or magnetic resonance imaging (MRI) do not show high sensitivity and specificity in the diagnosis of micrometastases < 1 cm [22]. While the diagnosis of metastasis is important for staging, identifying metastasis risk factors is also of great significance for precision clinical treatment. With the development of medical technology, several treatment methods, including surgery, active chemotherapy, and stereotactic radiotherapy, have been applied to the clinical practice of metastatic sites and have proven effective [23]. Preclinical studies have shown that blocking PD-1 can inhibit tumor growth and even reduce metastasis, which may provide a new direction for treating LM in patients with ovarian cancer.

The performance of traditional logistic regression prediction is unsatisfactory. Therefore, there is an urgent need to develop more accurate and practical predictive models based on clinical-pathological feature data. This population-based study explored the relationship between LM and risk factors in patients with ovarian cancer, which is essential for designing effective treatment strategies. To the best of our knowledge, this is the first study to use machine learning algorithms to study the risk factors associated with LM in patients with ovarian cancer.

This study used the XGBoost algorithm and SEER database to generate a risk model based on clinical and tumor characteristics, thereby predicting the risk of lung metastasis in newly diagnosed patients with ovarian cancer. We found that the most important factors were age, laterality, histological type, grade, marital status, AJCC T stage, AJCC N stage, tumor size, and liver metastasis. Previous univariate logistic regression analysis showed that age > 61 years, bilateral tumors, low-grade differentiation, and higher T and N stages are risk factors related to lung metastasis in patients with ovarian cancer [9, 11]. Previous studies have found that late-stage, high-grade, and lymph node involvement are important risk factors related to distant metastasis [24]. Our research confirmed this point. The importance of these factors lies at the forefront of the factors influencing ovarian cancer and lung metastasis. An autopsy study of 428 patients with ovarian cancer showed that for ovarian epithelial tumors, lymph node metastasis and intraperitoneal metastasis were related to distant metastasis to the lungs [25]. Aure et al. observed that serous cancer spreads to the upper abdomen [26]. Knapp and Friedman observed differences in the frequency of lymph node metastasis of different histological types during laparotomy or lymphangiography [27]. They found that with an increase in histological grade, there was a significant increase in retroperitoneal lymph node metastasis during open surgery, and the frequency of lymph node metastasis around the aorta and pelvis increased [28]. In a study of 1242 women based on the SEER database, we found that low-grade serous, endometrioid, and mucous histological lymph node metastasis rates were lower than those of high-grade tumors. Lymph node metastasis is highly related to distant metastases such as lung metastasis. Large-sample studies of bone metastases from ovarian cancer also believe that bone metastasis tends to occur in high-grade rather than low-grade cases and has a higher probability in nonserous ovarian cancer [29]. Therefore, tumor grade and histological type may affect the lung metastasis rate of ovarian cancer. This study also confirmed that the histological type and grade ranked third and fourth among all influencing factors. A study of 19,692 patients from the SEER database found that tumor size was an independent risk factor for lymph node metastasis in endometrioid endometrial cancer [30]. Previous studies have not found a relationship between tumor size and lung metastasis in patients with ovarian cancer. Our research suggests that tumors have an impact on the occurrence of lung metastasis in patients with ovarian cancer, but this contribution is not strong.

In recent years, various machine-learning algorithms have emerged. They have been developed to predict results by “learning” from data. They were studied to predict the pathological diagnosis and survival prognosis of ovarian cancer [31]. XGBoost is based on decision trees and has been found to be the best algorithm for machine learning and prediction competitions hosted by http://Kaggle.com/. Owing to its high accuracy and performance, algorithmic machine learning based on XGBoost has received increasing attention and is often used as a competitive alternative to regression analysis. Xu et al. found that a higher T stage, N1 stage, advanced tumor grade, and elevated cancer antigen 125 levels were associated with a higher risk of lung metastases at the time of diagnosis of ovarian cancer EOC; however, a model that facilitated clinical application was not constructed [10]. Cao and Yang constructed a model using logistic regression to screen for lung metastasis risk factors. The results showed that LM positively correlated with the T/N stage, bone metastasis, liver metastasis, and chemotherapy. However, it includes a few variables, and the evaluation of the model is insufficient [9]. Yuan et al. evaluated AJCC T and N stage, bone metastases, brain metastases, and liver metastases as predictors of synchronous lung metastases using logistic regression, and the accuracy of the model was not high; the AUC and sensitivity of the logistic regression model were only 0.761 and 0.474, respectively [11]. ML handles overfitting, imbalanced data distributions, and so on better than traditional statistical methods [32]. In this study, the XGBoost model of lung metastasis in patients with ovarian cancer has an AUC of 0.843 and a sensitivity of 1.000. The prediction performance of the XGBoost algorithm is significantly higher than that of logistics regression.

This is the first model to predict lung metastasis in patients with ovarian cancer, based on standard clinicopathological features and a novel AI algorithm. It extends the nomogram model based on logistic regression, which other researchers have often used. Our model performed exceptionally well in predicting lung metastasis in patients with ovarian cancer and could potentially assist clinicians in making more accurate and personalized medical decisions. However, this study has some limitations. First, the model is based on machine and deep learning algorithms; therefore, it might be difficult to clinically explain the important features selected by the model. Further work is required to transform this algorithm into a convenient scoring system for clinical use. Second, the SEER database records information at the time of initial diagnosis; therefore, it is impossible to analyze lung metastases that occur in the disease's later stages.

## 5. Conclusion

The XGBoost method is more effective and accurate than logistic regression in predicting the occurrence of lung metastases in patients with ovarian cancer. Creating user-friendly programs in mobile electronic devices based on the XGBoost algorithm will help evaluate patients with ovarian cancer at risk of lung metastasis to make appropriate treatments in the future.

## Figures and Tables

**Figure 1:** Flowchart of patient selection.

**Figure 2:** Features selected using XGBoost and the corresponding variable importance score. The *X*-axis indicates the importance score, which is the relative number of variables used to distribute the data, and the *Y*-axis indicates the top 14 weighted variables.

**Figure 3:** Receiver operating characteristic (ROC) curve. For the XGBoost model, the area under the curve (AUC) is 0.843.

**Table 1:** Demographical and clinical characteristics between patients with lung metastases and patients without lung metastases.

Variables	All patients (*N* = 16059)	Patients with lung metastases (*N* = 411)	Patients without lung metastases (*N* = 15648)	*P* value
Age	59 (50-68)	62 (54-59)	59 (50-68)	<0.001
Race				0.192
White	13223 (82.3%)	327 (79.6%)	12896 (82.4%)	
Black	1057 (6.6%)	33 (8.0%)	1024 (6.5%)	
Other (American Indian/AK Native, Asian/Pacific Islander)	1711 (10.7%)	51 (12.4%)	1660 (10.6%)	
Unknown	68 (0.4%)	0 (0.0%)	68 (0.4%)	
Marital status				0.170
Unmarried	3377 (21.0%)	84 (20.4%)	3293 (21.0%)	
Married	8549 (53.2%)	226 (55.0%)	8323 (53.2%)	
Separated	3486 (21.7%)	93 (22.6%)	3393 (21.7%)	
Unknown	647 (4.0%)	8 (1.9%)	639 (4.1%)	
Insurance status				0.932
Uninsured	561 (3.5%)	13 (3.2%)	548 (3.5%)	
Insured	15337 (95.5%)	394 (95.9%)	14943 (95.5%)	
Unknown	161 (1.0%)	4 (1.0%)	157 (1.0%)	
Tumor size				0.139
<2 cm	1305 (8.1%)	40 (9.7%)	1265 (8.1%)	
2-5 cm	2678 (16.7%)	79 (19.2%)	2678 (16.7%)	
>5 cm	12076 (75.2%)	292 (71.0%)	12076 (75.2%)	
Laterality				<0.001
Left	4947 (30.8%)	107 (26.0%)	4840 (30.9%)	
Right	5109 (31.8%)	92 (22.4%)	5017 (32.1%)	
Bilateral	6003 (37.4%)	212 (51.6%)	5791 (37.0%)	
Grade				<0.001
Well differentiated	2011 (12.5%)	9 (2.2%)	2002 (12.8%)	
Moderate differentiated	2758 (17.2%)	35 (8.5%)	2723 (17.4%)	
Poor differentiated	6395 (39.8%)	200 (48.7%)	6195 (39.6%)	
Undifferentiated	4895 (30.5%)	167 (40.6%)	472 (30.2%)	
AJCC T stage				<0.001
T1	5500 (34.2%)	28 (6.8%)	5472 (35.0%)	
T2	2552 (15.9%)	51 (12.4%)	2501 (16.0%)	
T3	8007 (49.9%)	332 (80.8%)	7675 (49.0%)	
AJCC N stage				<0.001
N0	12514 (78.0%)	239 (58.2%)	12275 (78.4%)	
N1	3545 (22.1%)	172 (41.8%)	3373 (21.6%)	
Bone metastasis				<0.001
Yes	54 (0.3%)	17 (4.1%)	37 (0.2%)	
No	16005 (99.7%)	394 (95.9%)	15611 (99.8%)	
Brain metastasis				0.017
Yes	15 (0.1%)	4 (1.0%)	11 (0.1%)	
No	16044 (99.9%)	407 (99.0%)	15637 (99.9%)	
Liver metastasis				<0.001
Yes	572 (3.6%)	97 (23.6%)	475 (3.0%)	
No	15487 (97.4%)	314 (76.4%)	15173 (97.0%)	
Histological type				<0.001
Serous	8644 (53.8%)	289 (70.3%)	8355 (53.4%)	
Endometrioid	2367 (14.7%)	20 (4.9%)	2347 (15.0%)	
Mucinous	1071 (6.7%)	6 (1.5%)	1065 (6.8%)	
Clear cell	1124 (7.0%)	11 (2.7%)	1113 (7.1%)	
Carcinosarcoma	515 (3.2%)	22 (5.4%)	493 (3.2%)	
Malignant Brenner	18 (0.1%)	0 (0.0%)	18 (0.1%)	
Carcinoma, NOS	516 (3.2%)	26 (6.3%)	490 (3.1%)	
Mixed	1140 (7.1%)	23 (5.6%)	1117 (7.1%)	
Other	664 (4.1%)	14 (3.4%)	650 (4.2%)	

## Data Availability

https://seer.cancer.gov/data/ is available for the Surveillance, Epidemiology, and End Results Program database.
